RETRACTED

# Evaluation of Teachers' Educational Technology Ability Based on Fuzzy Clustering Generalized Regression Neural Network

**DOI:** 10.1155/2021/1867723

**Published:** 2021-09-13

**Authors:** Jie Zhao, Honghai Guan, Changpeng Lu, Yushu Zheng

**Affiliations:** ^1^School of Computer and Information Technology, Mudanjiang normal University, Mudanjiang 157011, Heilongjiang, China; ^2^School of Education Science, Mudanjiang normal University, Mudanjiang 157011, Heilongjiang, China; ^3^College of Information Engineering, Heilongjiang Agricultural Economy Vocational College, Mudanjiang 157041, Heilongjiang, China

## Abstract

The improvement of teachers' educational technology ability is one of the main methods to improve the management efficiency of colleges and universities in China, and the scientific evaluation of teachers' ability is of great significance. In view of this, this study proposes an evaluation model of teachers' educational technology ability based on the fuzzy clustering generalized regression neural network. Firstly, the comprehensive evaluation structure system of teachers' educational technology ability is constructed, and then the prediction method of teachers' ability based on fuzzy clustering algorithm is analysed. On this basis, the optimization prediction method of fuzzy clustering generalized regression neural network is proposed. Finally, the application effect of fuzzy clustering generalized regression neural network in the evaluation of teachers' educational technology ability is analysed. The results show that the evaluation system of teachers' educational technology ability proposed in this study is scientific and reasonable; fuzzy clustering generalized regression neural network model can better accurately predict the ability of teachers' educational technology and can quickly realize global optimization. According to the fitness analysis results of the fuzzy clustering generalized regression neural network model, the model converges after the 20th iteration and the fitness value remains about 1.45. Therefore, the fuzzy clustering generalized regression neural network has stronger adaptability and has been optimized to a certain extent. The average evaluation accuracy of fuzzy clustering generalized regression neural network model is 98.44%, and the evaluation results of the model are better than other algorithms. It is hoped that this study can provide some reference value for the evaluation of teachers' educational technology ability in colleges and universities in China.

## 1. Introduction

Carrying out the evaluation of teachers' educational technology ability is one of the necessary ways to strengthen the management efficiency of colleges and universities in China, and it is also the main method to deepen the internal management system of colleges and universities. Without scientific and effective evaluation and management of teachers' educational technology ability, universities cannot achieve sustainable development [1]. The evaluation standard system of teachers' teaching ability is the main basis for colleges and universities to manage teachers. In order to effectively enhance the comprehensive competitiveness of colleges and universities in the field of education, it is very necessary to build a set of evaluation system of teachers' educational technology ability suitable for their own development [2]. However, there are many disadvantages in the past evaluation methods, which are mainly reflected in the heavy workload of questionnaire survey, one person instead of many people for questionnaire survey, and the incomplete evaluation system [3]. Therefore, colleges and universities are in urgent need of a scientific and fair evaluation method of teachers' educational ability in order to give correct guidance and encouragement to teachers. In recent years, there are more and more methods to evaluate the educational technology ability of university teachers, such as analytic hierarchy process, statistics, fuzzy c-means algorithm (FCM), and other methods, which make teachers' ability get quantitative and qualitative evaluation [4]. Among them, FCM is a traditional soft clustering algorithm, which can better deal with low dimensional data, allow the overlapping of several clusters, allow the existence of fuzzy boundaries, and can better predict the data structure [5]. However, FCM is a local search optimization algorithm. In order to effectively improve the accuracy of the evaluation of teachers' educational technology ability, this study introduces the combination of general regression neural network (GRNN) and FCM. GRNN is a branch of radial basis function neural network (RBF), which is a nonlinear regression feedforward neural network. The algorithm has the advantages of small amount of calculation and fast convergence and is widely used in larger fields [6].

RETRACTED

With the development of fuzzy clustering algorithm and generalized regression neural network algorithm, these two algorithms have become popular algorithms in algorithm model in recent years. Dai et al. used genetic algorithm (GA) optimization method, *k*-means method, and several soft computing (SC) models to better estimate land subsidence and proposed and evaluated genetic algorithm, *k*-nearest neighbor method, and ordered weighted average method (OWA) based on orness method and orlike method [7]. The results show that the method based on fusion is superior to the single method in predicting land subsidence rate. Eun-Hu and Sung proposed a fuzzy clustering-based ensemble neural networks (FCENNS) classifier, which combines probability model with learning mechanism, develops the design method of neural network classifier based on fuzzy clustering, and improves the learning method of fuzzy clustering neural network [8]. The proposed FCENNS classifier considers cross entropy error function to improve learning and generalization ability. Hsieh et al. proposed a new single index fuzzy neural network model, which replaced the output nodes of the network with (nonparametric) the single index model. The simulation results show that the proposed model has good fitting ability to the existing data [9]. Wu et al. proposed a new data-driven crude oil price prediction method, using Google trend and online media text mining. Convolutional neural network (CNN) is used to automatically extract text features from online crude oil news to illustrate the explanatory power of text features on crude oil price prediction [10]. The average absolute percentage errors of crude oil price prediction in the two cases are 0.0571 and 0.0459, respectively, indicating that the complementary relationship between news headlines and Google trend is conducive to fairly accurate crude oil price prediction. In order to make a useful analysis of brain activity, different variants of artificial neural network (ANS) and adaptive neuro fuzzy inference system (ANFIS) were compared. Generalized regression neural network (GRNN) with the minimum variance and 90% average accuracy exceeds eight network structures. In ANFIS model, fuzzy c-means model has the best overall performance, with an average accuracy of 95.45%, followed by subtractive clustering, with an average accuracy of 94% [11]. Wu et al. collected a large number of online oil news and automatically extracted relevant information using convolutional neural network, including oil price, oil production, oil consumption, and oil inventory. 8548 news headlines were collected in four different cases. The experimental results show that social media information is helpful to predict oil price, oil production, and oil consumption. During COVID-19 coronavirus disease, the average absolute percentage errors were 0.0717, 0.0144, and 0.0168, respectively. Marketers must consider the impact of social media information on oil or similar markets when coronavirus disease breaks out in 2019 [12]. Bansal et al. introduced Mahalanobis distance, which involves the covariance matrix between variables, and gave the extension of this distance to fuzzy frame. Generally, aspheric clusters that cannot be identified by Euclidean distance can be identified by the suggested distance [13]. Parwez et al. found the web-personalized fuzzy clustering algorithm of configuration files through experimental evaluation. The fuzzy clustering algorithm can cluster users' behaviours according to their interest and can be used for overlapping. The results show that this clustering method can generate website access log data through mining. Classification is a convolutional neural network (CNN), which is very useful for classification of objects with similar functions [14]. Entezami et al. compared the performance of the generalized regression neural network (ANN), artificial neural network (ANN), and adaptive neuro fuzzy disturbance system (ANFIS) in hydraulic parameter estimation, that is, storage coefficient and transfer coefficient of confined aquifer. The results show that, among all the intelligent prediction models used to estimate the hydraulic parameters of confined aquifer, ANFIS is more accurate than other models and requires less calculation time, so it can be selected as the best model for aquifer parameter estimation [15]. Zhao et al. designed a tissue segmentation method for PET/MR images based on TFC-BPNN-leverage tissue segmentation (TFC-NN-TSAC) by combining TFC and BPNN. The results show that the proposed TFC-NN-TSAC method has good tissue segmentation performance for Dixon-based MR data and good communication performance for PET images [16]. Tang proposed a self-organizing neural network-based evaluation method of westerly music form. Fuzzy clustering method was used to classify and evaluate the artistic expression of westerly music [17]. Finally, an example is given to verify the effectiveness of the proposed self-organizing neural model in the evaluation of Xifeng music form. Bodyanskiy et al. proposed an architecture of multilayer kernel clustering neuro fuzzy system and its self-learning algorithm, which can be used to recover overlapping clusters when feeding online [18]. The designed system is based on *t*. Kohonen's self-organizing mapping allows the recovery of linear and nonseparated data classes, processes information online, is not affected by dimensional constraints, and is easy to implement.

RETRACTED

To sum up, a large number of scholars have studied and applied fuzzy clustering and generalized regression neural network in various fields. In view of this, this study proposes an evaluation model of teachers' educational technology ability based on the fuzzy clustering generalized regression neural network and realizes the scientific evaluation method based on artificial intelligence technology, so as to provide some reference for the evaluation and prediction of teachers' ability. The specific technical route and process of this study are shown in Figure 1.

## 2. Fuzzy Clustering Generalized Regression Neural Network Evaluation Method

### 2.1. The Comprehensive Evaluation Structure System of Teachers' Educational Technology Ability

This study takes the data of a university in Chengdu from 2016 to 2020 as the sample to analyse the comprehensive level of teachers' teaching and uses the analytic hierarchy process (AHP) to construct the evaluation standard of teachers' teaching ability, as shown in Table 1.

In the hierarchical structure model of this study, there are five elements in the middle layer, namely, teachers' quality, teaching attitude, teaching content, teaching method, and teaching effect. The bottom level includes 18 indicators, including clear educational objectives, solid professional knowledge, teaching and explanation level, and patient and positive counselling and answering. The evaluation results of the index system of teachers' educational technology ability are taken as the output of the prediction model below, and the evaluation level is shown in Table 2.

### 2.2. Prediction Method of Teachers' Ability Based on Fuzzy Clustering Algorithm

Fuzzy c-means clustering (FCM) algorithm is an optimized hard c-means clustering algorithm. The algorithm mainly selects multiple clustering centers in Euclidean space, assigns each data point to each clustering center through a certain rule membership, and then iterates the iteration center. To minimize the weighted sum of the distance from each data point to each cluster center and the membership value [19]. Set the space *X*={*x*_1_, *x*_2_,…, *x*_*n*_} and divide the points of *n* data samples into *c* types, where 2 ≤ *c* ≤ *n* and {*A*_1_, *A*_2_,…, *A*_*c*_} can be used to represent the corresponding *c* types, *U* is the similarity classification matrix, the cluster center of each type can be represented as *V*={*v*_1_, *v*_2_,…, *v*_*c*_}, and the membership degree of sample *A*_*k*_ to type *x*_*i*_ is *u*_*ik*_. Therefore, the objective function *J*(*U*, *V*) of FCM is shown as follows:

(1) $$\begin{array}{c} J\left(U,V\right)=\sum_{i=1}^{n}\sum_{k=1}^{c}{\left(u_{ik}\right)}^{2}{\left({\text{d}}_{ik}\right)}^{2}. \end{array}$$

Here, *m* is the fuzzy index, *m* ∈ [1, *∞*). Based on previous research results, the value of this study is 2; ∑_*k*=1_^*c*^*u*_*ik*_=1, *u*_*ik*_ ∈ [0,1], (d_*ik*_)^2^=‖*x*_*k*_ − *v*_*i*_‖^2^, and d_*ik*_ are Euclidean distance between cluster center *v*_*i*_ and sample point *x*_*k*_ [20]. In order to minimize the value of *J*(*U*, *V*) to achieve the optimal classification effect, the clustering center matrix *v*_*i*_ and *u*_*ik*_ can be obtained by using Lagrange function as follows:

(2) $$\begin{array}{c} u_{ik}={\left(\sum_{j=1}^{c}{\left(\frac{d_{ik}}{d_{jk}}\right)}^{2/m-1}\right)}^{-1},\;1\leq i\leq c,\;1\leq k\leq n, \end{array}$$

(3) $$\begin{array}{c} v_{i}=\frac{\sum_{k=1}^{n}{\left(u_{ik}\right)}^{m}x_{k}}{\sum_{k=1}^{n}{\left(u_{ik}\right)}^{m}},\;1\leq i\leq c. \end{array}$$

FCM algorithm steps can be divided into four steps: one is to set the number of clusters *c*, fuzzy index *m*, the number of iterations and the maximum number of iterations *a* and *a*_max_, iteration stop error *ε*, initialize cluster center *V*^(0)^, and initialize membership matrix *U*^(0)^. The second step is to calculate *u*_*ik*_. The third step is to update *v*_*i*_. In the fourth step, a matrix norm is selected to compare the membership matrix before and after iteration ‖*U*^(*t*+1)^ − *U*^(*t*)^‖ ≤ *ε*. If the condition is not satisfied, return to the second step to continue the iteration [21]. Among them, the value of cluster number *c* needs to be set in advance. In order to avoid the error caused by managers' subjective experience, this study uses the cluster validity function to determine the *c* value. The expression of the cluster validity function is shown as follows:

(4) $$\begin{array}{c} R\left(U;c\right)=\overset{c}{\underset{j=1}{\text{max}}}\overset{c}{\underset{k=1,k\neq j}{\text{max}}}R_{jk}\left(U;c\right). \end{array}$$

Here, *R*_*jk*_ is the fuzzy correlation degree of class *j* and *k* and the expression of *R*_*jk*_ is shown as follows:

(5) $$\begin{array}{c} R_{jk}=\frac{\sum_{h=1}^{n}u_{hj}^{m/2}u_{hk}^{m/2}\left\|x_{h}-v_{j}\right\|\left\|x_{h}-v_{k}\right\|}{{\left(\sum_{h=1}^{n}u_{hj}^{m}{\left\|x_{h}-v_{j}\right\|}^{2}\right)}^{1/2}{\left(\sum_{h=1}^{n}u_{hk}^{m}{\left\|x_{h}-v_{k}\right\|}^{2}\right)}^{1/2}}. \end{array}$$

In formula (5), ‖*x*_*h*_ − *v*_*k*_‖ and ‖*x*_*h*_ − *v*_*j*_‖ represent the cluster center and the distance between the cluster center *v*_*j*_ and the sample point *v*_*k*_, respectively. *u*_*hk*_ and *u*_*hj*_ denote the membership degree of *x*_*h*_ belonging to class *k* and class *j*, respectively. If the fuzzy correlation between different classes is smaller, the classification effect is better. Let the optimal finite set of *U* be Ω_*c*_, then the optimal efficient clustering AA satisfies the condition as follows:

(6) $$\begin{array}{c} R\left(U^{*};c^{*}\right)=\underset{c}{\max}\left\{\underset{Kc}{\max}R\left(U;c\right)\right\}. \end{array}$$

Here, *c*^*∗*^ represents the optimal number of categories.

RETRACTED

It is necessary to ensure the accuracy of test data collection to introduce FCM algorithm into the teacher ability prediction method. In order to guarantee the ability of clustering in prediction, the sample data set has a very low proportion of abnormal data and has a high amount of normal data, which is usually about 98%. The size of the classifier can judge the abnormal class and normal class to distinguish the clustering results. The small cluster usually has a low amount of data, which is represented as the clustering of abnormal data. However, the large cluster is opposite to the small cluster, which means clustering of normal data. Take out the test data set one by one and match the class center of the marked class. If the matching degree is low, it means that the output is abnormal. If the matching degree is high, the data is output normally [22]. Therefore, the FCM algorithm is designed here. The design includes three stages: clustering, labeling, and matching, as shown in Figure 2.

## 3. Fuzzy Clustering Generalized Regression Neural Network Optimization Prediction Method

FCM is a local search optimization algorithm, which mainly uses the random allocation mode to select the initial cluster center, resulting in a greater impact on the stability of the algorithm. Therefore, the execution results of each algorithm may be different, so that the FCM algorithm will converge at the local extremum point and eventually fall into the local optimal solution [23]. Therefore, this study proposes to use the generalized regression neural network (GRNN) combined with FCM to predict teachers' educational ability. GRNN algorithm belongs to the branch of radial basis function neural network (RBF), which is a kind of the nonlinear regression feedforward neural network. The algorithm has the advantages of small amount of calculation and fast convergence and is widely used in larger fields [24, 25]. The GRNN algorithm model is shown in Figure 3.

Firstly, input *m* dimension, input variable *X*=[*x*_1_, *x*_2_,…,*x*_*m*_]^*T*^, and the number of neurons in input layer is the same as *m*. After the data arrive at the pattern layer, the number of neurons in the pattern layer is equal to the number of samples *n*, and they correspond to each other. Then, it can be assumed that there exists

(7) $$\begin{array}{c} D_{i}^{2}={\left(X-X_{i}\right)}^{T}\left(X-X_{i}\right). \end{array}$$

Here, *X*_*i*_ is the *i* learning samples of the *m* dimensional neuron. In the model layer, the activation kernel function with Gauss function is *i*, and the transfer function is shown as follows:

(8) $$\begin{array}{c} p_{i}=\exp\left[-\frac{D_{i}^{2}}{2\sigma^{2}}\right],\;i=1,2,\ldots ,n. \end{array}$$

Here, *σ* represents the smoothing parameter. The summation layer of GRNN has two different types of neuron summation processes as follows:

(9) $$\begin{array}{c} S_{D}=\sum_{i}^{n}p_{i}, \end{array}$$

(10) $$\begin{array}{c} S_{N}=\sum_{i}^{n}Y_{i}p_{i}. \end{array}$$

Among them, the connection weight between each neuron is 1. In the output layer, the predicted value of GRNN model is obtained as follows:

(11) $$\begin{array}{c} \overset{\wedge }{Y}=\frac{S_{N}}{S_{D}}. \end{array}$$

The GRNN model applies the predictive value of nonindependent variables in regression analysis, which is the input value relative to independent variables. For independent variable *X* and nonindependent variable *Y*, the output variable AA with the maximum probability value is calculated. Let *f*(*X*, *Y*) be the joint probability density function of variables *X* and *Y*, so the calculation of conditional mean is shown as follows:

(12) $$\begin{array}{c} \overset{\wedge }{Y}=E\left[Y|X\right]=\frac{\int_{-\infty }^{+\infty }Yf\left(X,Y\right)\text{d}y}{\int_{-\infty }^{+\infty }f\left(X,Y\right)\text{d}y}. \end{array}$$

The nonparametric samples are used to estimate *X* and *Y* observation samples. The calculation of *f*(*X*, *Y*) is shown as follows:

(13) $$\begin{array}{c} \overset{\wedge }{Y}\left(X,Y\right)=\frac{1}{{\left(2\pi \right)}^{\left(m+1\right)/2}\sigma^{m+1}n}\times \sum_{i=1}^{n}\exp\left[-\frac{D_{i}^{2}}{2\sigma^{2}}\right]\exp\left[-\frac{\left(Y-Y_{i}\right)}{2\sigma^{2}}\right], \end{array}$$

(14) $$\begin{array}{c} Y\left(X\right)=\frac{\sum_{i=1}^{n}\left[\exp\left(-\left(D_{i}^{2}/2\sigma^{2}\right)\right)\right]\int_{-\infty }^{+\infty }Y_{j}\exp\left[-\left(Y-Y_{i}\right)/2\sigma^{2}\right]\text{d}y}{\sum_{j=1}^{n}\left[\exp\left(-\left(D_{j}^{2}/2\sigma^{2}\right)\right)\right]\int_{-\infty }^{+\infty }Y_{j}\exp\left[-\left(Y-j\right)/2\sigma^{2}\right]\text{d}y}. \end{array}$$

Among them, ∫_−*∞*_^+*∞*^*xe*^−*x*^2^^d*x*=0, set parameter variables *z*=*Y* − *Y*_*i*_. Then, we can get

(15) $$\begin{array}{c} \int_{-\infty }^{+\infty }Y_{i}\exp\left[-\frac{\left(Y-Y_{i}\right)}{2\sigma^{2}}\right]\text{d}y=Y_{i}\int_{-\infty }^{+\infty }\exp\left(-\frac{z^{2}}{2\sigma^{2}}\right)\text{d}z, \end{array}$$

(16) $$\begin{array}{c} \int_{-\infty }^{+\infty }\exp\left[-\frac{\left(Y-Y_{i}\right)}{2\sigma^{2}}\right]dy=\frac{\sum_{i=1}^{n}\left[\exp\left(-\left(D_{i}^{2}/2\sigma^{2}\right)\right)\right]\int_{-\infty }^{+\infty }Y_{i}\exp\left[-\left(Y-Y_{i}\right)/2\sigma^{2}\right]\text{d}y}{\sum_{j=1}^{n}\left[\exp\left(-\left(D_{j}^{2}/2\sigma^{2}\right)\right)\right]\int_{-\infty }^{+\infty }Y_{j}\exp\left[-\left(Y-j\right)/2\sigma^{2}\right]\text{d}y} \end{array}$$

If the training samples are fixed, the essence of GRNN algorithm becomes the determination process of smoothing parameter *σ*. If the smoothing parameter approaches infinity, *Y*(*X*) is the mean value of all training samples; while when the smoothing parameter approaches zero, the training samples are basically consistent with the estimated value. Then, the GRNN is optimized by chaos optimization algorithm to prevent the algorithm from falling into local minimization, so as to improve the search efficiency as follows:

(17) $$\begin{array}{c} Y_{n+1}=\mu y_{n}\left(1-y_{n}\right),\;n=0,1,2,\ldots ,0\leq \mu \leq 4. \end{array}$$

Here, *μ* represents the control parameters. Generally, GRNN has two major defects. One is that when the training sample increases, the result will be too large, which makes the model calculation more complex and has a great impact on the calculation efficiency. Second, the smoothing parameters will affect the accuracy of the model calculation, and GRNN usually only uses a single smoothing parameter to calculate, so the calculation results are not accurate enough. Therefore, this study combines FCM algorithm with GRNN algorithm to get a new evaluation model. The optimized model is shown in Figure 4.

RETRACTED

FCM algorithm combines the basic idea of GRNN algorithm. Firstly, FCM is used to cluster historical data [26]. After the clustering process is completed, multiple samples in the clustering are selected as training samples, and GRNN model is trained. The dynamic model is optimized by chaotic variables, and the training optimization process is repeated. When the calculation error is reduced to controllable range, the whole training iteration is completed [27].

## 4. Application Effect Analysis of Fuzzy Clustering Generalized Regression Neural Network

The evaluation indexes of teachers' educational technology ability proposed in this study are all positive indexes, and the weight of the evaluation index system is determined according to the steps of the entropy method [28]. The results are shown in Table 3.

This study finally determined 1000 groups of experimental data samples, 900 groups of data samples as model training, in order to get the optimal model, and the other 100 groups as test samples; some of the test data are shown in Table 4.

MATLAB is used to realize the simulation experiment of the evaluation of teachers' educational technology ability based on the fuzzy clustering generalized regression neural network. 100 test sets are predicted and evaluated, and the results are shown in Figure 5. It can be seen from Figure 5 that the root mean square error of the first 30 iterations of the teacher ability prediction model based on fuzzy clustering algorithm decreases rapidly, converges after the 87th iteration, and converges at 8.6066*e *−* *08, during which the 31st to 80th iterations are relatively slow [29]. The first iteration speed of the fuzzy clustering generalized regression neural network model is faster, but it is slower in the second to the eighth iteration. After the ninth iteration, the mean square error converges to 3.3893*e *−* *12, which improves the convergence accuracy and speed of the model. The convergence accuracy is improved by 100%, and the convergence speed is improved by 79.35%. The results show that the fuzzy clustering generalized regression neural network model can better predict the ability of teachers' educational technology [30].

RETRACTED

Compare the error sum of square of the fuzzy clustering generalized regression neural network and the error sum of the fuzzy clustering algorithm. The results are shown in Figure 6. The convergence speed of the 10th iteration of the minimum error and average error of fuzzy clustering algorithm is faster, the 10th to 25th iterations are slower, and the error remains about 0.9 after the 25th iteration. The fuzzy clustering generalized regression neural network converges after only 6 iterations, the sum of square error converges to 0.19, the average sum of square error reduces by 78.81%, and the relative convergence speed increases by 77.21%. Therefore, the fuzzy clustering generalized regression neural network can quickly achieve global optimization.

Figure 7(a) shows that the best stage of fuzzy clustering algorithm and the fastest convergence speed of average fitness is before the 20th generation, the 40th to 60th iterations are relatively slow, and the convergence is stable after the 67th iteration, and the fitness value remains about 0.85.  Figure 7(b) shows the results of fitness analysis of the fuzzy clustering generalized regression neural network model. The model converges after the 20th iteration, and the fitness value remains at about 1.45. Therefore, the fuzzy clustering generalized regression neural network has stronger adaptability and has been optimized to a certain extent.

The comparison results of model evaluation accuracy are shown in Table 5. The results show that the average evaluation accuracy of the BP neural network, fuzzy clustering algorithm model, genetic algorithm (GA) optimized BP neural network, and fuzzy clustering generalized regression neural network model is 84.37%, 91.74%, 92.63%, and 98.44%, respectively, and FCM-GRNN is increased by 14.07%, 6.70%, and 5.18% respectively. The time consumption of each method is 16.92s, 13.03s, 11.65s, and 6.15s, respectively, and the FCM-GRNN is increased by 10.77%, 6.88s, and 5.5s, respectively. Therefore, the evaluation result of the fuzzy clustering generalized regression neural network model is better.

RETRACTED

## 5. Conclusion

Aiming at the evaluation of college teachers' educational technology ability, this paper proposes an evaluation model of teachers' educational technology ability based on the fuzzy clustering generalized regression neural network and analyses the application effect of the model in the evaluation of teachers' educational technology ability. The evaluation system of teachers' educational technology ability proposed in this study is scientific and reasonable. Fuzzy clustering generalized regression neural network model can better accurately predict the ability of teachers' educational technology and can quickly realize global optimization. According to the fitness analysis results of the fuzzy clustering generalized regression neural network model, the model converges after the 20th iteration and the fitness value remains about 1.45. Therefore, the fuzzy clustering generalized regression neural network has stronger adaptability and has been optimized to a certain extent. The average evaluation accuracy of the fuzzy clustering generalized regression neural network model is 98.44%, and the evaluation results of the model are better than other algorithms. Therefore, the evaluation result of the fuzzy clustering generalized regression neural network model is better. Due to the limited ability, there is no further classification of the evaluation index system of teachers' ability, and more attention will be paid to this aspect in the future work.

## Figures and Tables

**Figure 1:** Specific technical route and process.

**Figure 2:** Design idea of FCM-based teacher ability prediction algorithm.

**Figure 3:** GRNN network model.

**Figure 4:** Flow chart of the improved generalized regression neural network learning algorithm.

**Figure 5:** Mean square error of the fuzzy clustering generalized regression neural network. (a) Prediction method of teachers' ability based on the fuzzy clustering algorithm. (b) Fuzzy clustering generalized regression neural network optimization prediction method.

**Figure 6:** Mean square error of the fuzzy clustering generalized regression neural network optimization prediction method. (a) The sum of square error of teachers' ability prediction method based on the fuzzy clustering algorithm. (b) The sum of square error fuzzy clustering generalized regression neural network.

**Figure 7:** Fuzzy clustering generalized regression neural network optimization prediction fitness. (a) Adaptability prediction of teachers' ability based on fuzzy clustering algorithm. (b) Fuzzy clustering generalized regression neural network optimization prediction fitness.

RETRACTED

**Table 1:** The comprehensive evaluation structure system of teachers' educational technology ability.

First level evaluation index	Secondary evaluation index	Index code
(A1) Quality of teachers	Clear education objectives	X1
	Solid professional knowledge	X2
	Teaching and explanation level	X3

(A2) Teaching attitude	Be patient and active in tutoring and answering questions	X4
	Teaching is serious and infectious	X5
	Rigorous attitude and continuous improvement	X6

(A3) Content of courses	The concept theory is accurate	X7
	Full content, ability oriented	X8
	Connecting with practice and paying attention to practice	X9
	Depth and breadth of professional knowledge	X10

(A4) Teaching method	Be good at inspiring and guiding thinking	X11
	Various ways and proper use	X12
	Pay attention to personality and teach according to their aptitude	X13
	Focus on stimulating innovation consciousness	X14

(A5) Teaching effectiveness	Improve self-study ability and interest in learning	X15
	Understanding and mastering of basic knowledge	X16
	Improve the ability of problem solving	X17
	Comprehensive quality and innovation ability	X18

**Table 2:** Each grade of evaluation result and its score range.

Serial number	Grade index	Score range
1	Excellent	[90, 100]
2	Good	[80, 89]
3	Secondary	[70, 79]
4	Pass	[60, 69]
5	Fail	[0, 59]

**Table 3:** Index weight of the teaching quality evaluation index system determined by the entropy method.

First level evaluation index	Secondary evaluation index	Index code	Weight
(A1) Quality of teachers	Clear education objectives	X1	0.05
	Solid professional knowledge	X2	0.07
	Teaching and explanation level	X3	0.08

(A2) Teaching attitude	Be patient and active in tutoring and answering questions	X4	0.06
	Teaching is serious and infectious	X5	0.06
	Rigorous attitude and continuous improvement	X6	0.05

(A3) Content of courses	The concept theory is accurate	X7	0.05
	Full content, ability oriented	X8	0.05
	Connecting with practice and paying attention to practice	X9	0.07
	Depth and breadth of professional knowledge	X10	0.06

(A4) Teaching method	Be good at inspiring and guiding thinking	X11	0.05
	Various ways and proper use	X12	0.06
	Pay attention to personality and teach according to their aptitude	X13	0.06
	Focus on stimulating innovation consciousness	X14	0.05

(A5) Teaching effectiveness	Improve self-study ability and interest in learning	X15	0.05
	Understanding and mastering of basic knowledge	X16	0.05
	Improve the ability of problem solving	X17	0.05
	Comprehensive quality and innovation ability	X18	0.05

**Table 4:** Some test input data.

Index code	1	2	3	4	5	6	7	8	9	10	......
X1	0.80	0.90	0.80	0.70	0.80	0.74	0.72	0.69	0.73	0.72	......
X2	0.80	0.78	0.83	0.83	0.78	0.76	0.81	0.73	0.80	0.73	......
X3	0.80	0.67	0.68	0.80	0.79	0.78	0.72	0.67	0.70	0.81	......
X4	0.73	0.74	0.80	0.70	0.80	0.89	0.72	0.72	0.70	0.77	......
X5	0.80	0.69	0.63	0.79	0.77	0.80	0.77	0.82	0.73	0.79	......
X6	0.74	0.70	0.69	0.77	0.78	0.77	0.79	0.78	0.77	0.85	......
X7	0.74	0.73	0.63	0.79	0.77	0.63	0.74	0.77	0.80	0.79	......
X8	0.73	0.80	0.77	0.70	0.73	0.76	0.80	0.81	0.85	0.77	......
X9	0.83	0.81	0.80	0.74	0.79	0.77	0.78	0.76	0.79	0.73	......
X10	0.77	0.70	0.77	0.67	0.61	0.81	0.79	0.79	0.81	0.76	......
X11	0.84	0.57	0.69	0.68	0.58	0.70	0.73	0.74	0.68	0.77	......
X12	0.79	0.63	0.63	0.81	0.69	0.74	0.77	0.77	0.76	0.80	......
X13	0.79	0.78	0.63	0.80	0.79	0.73	0.79	0.80	0.79	0.80	......
X14	0.83	0.75	0.64	0.83	0.79	0.80	0.82	0.77	0.70	0.73	......
X15	0.76	0.80	0.58	0.83	0.70	0.83	0.73	0.77	0.74	0.80	......
X16	0.81	0.51	0.66	0.69	0.79	0.69	0.77	0.87	0.80	0.81	......
X17	0.78	0.70	0.70	0.80	0.80	0.77	0.80	0.81	0.78	0.76	......
X18	0.66	0.68	0.59	0.67	0.74	0.68	0.74	0.77	0.81	0.77	......

RETRACTED

**Table 5:** Model performance comparison.

Model	Average evaluation accuracy (%)	Time (s)
BP neural network	84.37	16.92
FCM	91.74	13.03
GA-BP	92.63	11.65
FCM-GRNN	98.44	6.15

## Data Availability

The data used to support the findings of this study are available from the corresponding author upon request.
